# Plasma Neurofilament Light Chain Is Associated with Cognitive Impairment after Posterior Circulation Stroke

**DOI:** 10.1155/2022/2466982

**Published:** 2022-06-28

**Authors:** Lianyan Jiang, Zhiqiang Wang, Rongyu Wang, Mao Li, Yaodan Zhang, Dongdong Yang

**Affiliations:** ^1^Chengdu University of Traditional Chinese Medicine, Chengdu, China; ^2^Department of Neurology, Hospital of Chengdu University of Traditional Chinese Medicine, Chengdu, China; ^3^Department of Neurology, Chengdu BOE Hospital, Chengdu, China

## Abstract

**Background:**

Neurofilament light chain (NfL) is a biomarker for large-caliber axonal degeneration in the subcortex. The purpose of this research was to examine the relationship between plasma neurofilament light chain (pNfL) and cognitive impairment following a posterior circulation stroke.

**Methods:**

Patients over the age of 18 with their first-ever acute ischemic stroke (AIS) of the posterior cerebral circulation within 24 h of symptom onset were included from July 1, 2017, to December 31, 2019. Blood samples were collected within 48 h after the stroke. The Montreal Cognitive Assessment (MOCA) (MOCA < 26) was adopted to define poststroke cognitive impairment (PSCI) 90 days after stroke onset.

**Results:**

A total of 264 patients were analyzed in this research 101 (38.30%) patients were clinically diagnosed with PSCI. The PNfL concentration was significantly higher in the PSCI group compared with the non-PSCI group (*p* < 0.001). The pNfL concentration (OR 1.044; *p* < 0.001) remained to be a significant predictor for PSCI after a multivariable logistic regression analysis, even after adjusting for factors including age, sex, education background (OR 1.044; *p* < 0.001), baseline NIHSS, infarct volume, and TOAST classification (OR 1.035; *p* < 0.001). The diagnostic efficacy of pNfL concentration for PSCI was then explored with a ROC analysis. The optimum pNfL concentration threshold was 38.12 pg/ml, with a sensitivity of 78.20%, a specificity of 66.9%, and an AUC of 0.782 (*p* < 0.001).

**Conclusion:**

This research showed that pNfL concentration, independent of established conventional risk factors, could predict the cognitive impairment in 90 days following posterior circulation stroke.

## 1. Introduction

Stroke is the world's second most common cause of mortality and the main cause of adult disability [1]. Long-term or permanent impairment in cognitive function is common among stroke survivors [2]. One of the major consequences of a stroke is poststroke cognitive impairment (PSCI). Stroke is related to a five to eight times increase in the incidence of cognitive impairment [3]. Based on a recent study, the overall prevalence of PSCI in China is significant, reaching 80.97% [4]. PSCI patients suffer from a poor prognosis, which includes functional disability, death, and recurrent stroke [5, 6]. Therefore, early diagnosis of cognitive damage after a stroke is of great importance for the improvement of patients' life quality and prognosis. Biomarkers in circulating blood serum, plasma, and cerebrospinal fluid (CSF) of PSCI patients have been shown in several studies as important factors for the diagnosis and prediction of cognitive impairment in recent years [5]. Thus, more accurate biomarkers should be introduced for the better identification of individuals facing an increasing risk of PSCI promptly.

Neurofilaments are the major cytoskeletal constituents of neuronal cells. Neurofilament proteins are released into the extracellular environment by many pathological events that induce axonal injury [7, 8]. The NfL concentration released into the cerebrospinal fluid or peripheral blood is therefore regarded as a biomarker for axonal injury and neurodegeneration in a variety of neurological illnesses [2]. PNfL may better reflect the pathogenic rationale of PSCI compared with such previous blood markers as oxidative damage biomarkers, inflammatory factors, growth factors, and metabolic biomarkers [5]. Proteins can now be tested in serum and plasma other than in CSF, thanks to the development and implementation of new detection techniques. Serum NfL levels were found to be a significant predictor of clinical severity on admission and functional outcome at 3 months in stroke in recent investigations [9]. NfL in CSF and blood has been found to increase in the majority of neurodegenerative illnesses, including Alzheimer's disease (AD) and frontotemporal dementia (FTD), when compared with healthy controls according to a meta-analysis [10]. PNfL levels were related to cognitive domains and could serve as a predictor of functional improvement in the late period following a stroke [11]. PNfL was revealed to be a valuable marker for the prediction of the prognosis of nonspecific neurodegeneration and cognitive abnormalities [12]. However, there is a scarcity of data linking pNfL levels to PSCI. It is acknowledged that anterior circulation stroke can cause cognitive impairment, but many studies have shown that strokes caused by the inadequate blood supply in areas such as the brainstem and cerebellum of the posterior circulation can also lead to varying degrees of cognitive impairment. Previously, we found that pNfL concentration was an independent risk factor for PSCI 90 days after an anterior circulation stroke. In this research, we examined the relationship between pNfL and cognitive impairment after a posterior circulation stroke.

## 2. Materials and Methods

### 2.1. Study Design and Participants

The current research, conducted under the principles outlined in the Helsinki Declaration, was approved by the Medical Ethics Committee of the General Hospital of the Western Theater Command (No.71 2018ky06). A written informed consent form was signed by all participants or their relatives. Patients admitted to the Department of Neurology, Western Theater Command's General Hospital, were included in this research from July 1, 2017, to December 31, 2019. Patients included were those over the age of 18 who had experienced their first-ever AIS of the posterior circulation within 24 hours of symptom onset. AIS was validated based on the diagnostic criteria of the World Health Organization and was diagnosed as a posterior circulation ischemic stroke with brain computed tomography (CT) and magnetic resonance imaging (MRI). The following exclusion criteria were applied: (1) dementia or considerable cognitive impairment before the stroke (clinical diagnosis or previous treatment or self-reported cognitive impairment), mental disorders, or being unable to complete the cognitive exams; (2) major neurological illness other than stroke, for example, Parkinson's disease; and (3) autoimmune or haematologic illnesses, severe hepatic, renal, or thyroid problems, or cardiac failure.

The infarct volume (measured by MRI-DWI) and the National Institutes of Health and Stroke Scale (NIHSS) were employed to identify the severity of the stroke at the time of enrollment. The DWI infarct volumes were evaluated by two expert raters without knowing the clinical or laboratory outcomes and calculated based on slice thickness and infarction areas [13]. The Montreal Cognitive Assessment (MOCA) was used to measure changes in cognition at the 3-month follow-up by experienced psychiatrists who were blind to the clinical data (MOCA). This study adopted the English literal translation of the MOCA Beijing edition, and the following MOCA refers to the MOCA Beijing edition. A MOCA ＜ 26 points was used to define PSCI [14].

### 2.2. Blood Sampling and Biomarker Measurements

Blood samples were collected within 48 h after the stroke, and the stroke onset to blood sampling time was recorded. After being kept for 30 to 40 minutes at room temperature and centrifugated for 20 min at 3,000*g*, the samples were kept at −80°C. The single-molecule (Simoa) array was used to measure pNfL [15]. More detailed information about experimental methods can be found in our previous research [16].

### 2.3. Statistical Analysis

Based on MOCA scores, all participants were separated into PSCI and non-PSCI groups. The two subgroups' baseline characteristics were provided for contrast. Continuous variables were reported as means with standard deviation (SD) or medians with interquartile range (IQR), as appropriate. Categorical variables were presented in percentages. The nonparametric Spearman's rank correlation test was used to examine the correlations between clinical features of patients and plasma levels. The relationship between pNfL and PSCI was studied using a logistic regression model that was adjusted to the known factors. Variables that were shown to be significant in univariate analysis (*p* < 0.1) and other clinically significant variables were included as covariates in the regression analysis. The diagnostic accuracy of pNfL for PSCI was assessed with the receiver operating characteristic (ROC) curve analysis. A nonparametric technique was adopted to determine the best sensitivity and specificity. The Youden index was employed to find the cutoff value for the test that had the greatest discriminating power. SPSS 26 (IBM, Chicago, IL) was used for all of the analyses. *p* < 0.05 with two tails was considered to be significant.

## 3. Results

Table 1 shows the clinical background features and pNfL concentration for relevant patient categories. This study selected 310 posterior circulation stroke patients as participants. Twelve patients died within three months, eight patients had other central nervous system diseases, nine patients were unable to complete the cognitive assessments, seven patients withdrew consent or were lost to follow-up, and ten patients missed blood samples. Thus, 264 patients were finally enrolled in our research. Among participants [median age: 65 years (IQR, 51–73); male: 157 (59.47%)), 101 (38.30%) had a clinical diagnosis of PSCI; Based on the National Institutes of Health Stroke Scale, the median clinical severity was 5 points (NIHSS; IQR, 3–8), the median pNfL was 38.68 (IQR, 24.61–53.85) pg/ml, the median MOCA was 26.00 (IQR, 23.25–27.00), and the time interval from the index event to blood collection was kept the same among the groups. More details can be found in Table 1.

At the start of this research, there were no significant differences between the PSCI and non-PSCI groups in terms of education level, sex, smoking history, alcohol consumption, stroke type, and cardiovascular risk factors such as hypertension, diabetes mellitus, and atrial fibrillation (all *p*  >  0.05). After univariate analysis, the PSCI group, with older patients (median, 68 versus 62 years; *p*=0.005), had a greater infarction volume (median, 18.06 versus 11.05 mL, *p* < 0.001), more severe clinical impairments (median NIHSS 7 versus 4, *p*=0.001), and higher levels of homocysteine (HCY) (median, 16.45 versus 15.14 *μ*mol/L, *p*=0.042). Meanwhile, patients with PSCI were more likely to have hyperlipidemia (*p*=0.024). The time interval from stroke onset to blood collection, plasma high sensitivity C-reactive protein (Hs-CRP) level, and HbA1c levels were kept the same between the two groups (all *p*  >  0.05). PNfL was substantially greater in the PSCI group, at 49.54 pg/mL (IQR, 40.00–78.59) compared with the non-PSCI group, was at 30.12 pg/mL (IQR, 19.88–43.61), *p* < 0.001 (Table 1 and Figure 1).

In Spearman correlation analysis, pNfL levels were positively correlated with age (*r* = 0.146, *p*=0.017), the NIHSS score (*r* = 0.339, *p* < 0.001; Figure 2(a)), cerebral infarction volumes (*r* = 0.317, *p* < 0.001; Figure 2(b)), and the time for blood sampling (*r* = 0.377, *p* < 0.001; Figure 2(c)); pNfL levels were negatively correlated with the MOCA score (*r* = −0.323, *p* < 0.001; Figure 2(d)).

In the multivariate analysis, pNfL (OR, 1.044; 95% CI, 1.031–1.059; *p* < 0.001) remained to be significant predictor for PSCI, even after adjusting for age, sex, education level (OR, 1.044; 95% CI, 1.030–1.058; *p* < 0.001), baseline NIHSS, infarct volume, and TOAST classification(OR, 1.035; 95% CI, 1.019–1.051; *p* < 0.001). Details of information are shown in Table 2.

The Hosmer and Lemeshow (H–L) goodness of fit test indicated that the model was a good match to the data, with a *p* value of 0.343 (>0.05). The diagnostic efficacy of pNfL for PSCI was then analyzed with a ROC analysis. The best threshold was 38.12 pg/ml, which resulted in a sensitivity of 78.2% and a specificity of 66.9%, with an AUC of 0.782 (95% CI, 0.726–0.837; *p* < 0.001; Figure 3).

## 4. Discussion

The goal of this research was to explore if there was a relationship between pNfL levels in the acute phase of ischemic stroke (within 48 h of onset) and PSCI 90 days after a posterior circulation stroke even after adjusting for potential confounding factors. We discovered that the increase of pNfL was related with a greater risk of PSCI and that pNfL was an independent predictor for PSCI. PNfL levels were a reliable predictor of patients with PSCI. The level of pNfL within 48 hours of onset was revealed to be an independent risk factor for PSCI 90 days following an anterior circulation stroke in a previous study [16]. However, the prior study only observed patients who had an anterior circulation stroke and excluded those who had a posterior circulation stroke. This research made innovations for exploring the relationship between the cognitive impairment and pNfL levels after posterior circulation stroke.

PNfL is a potential biomarker that has been widely explored in the context of a variety of neurological illnesses. Axonal damage is indicated by an increase in pNfL levels, which can occur irrespective of the underlying pathophysiological process [10]. PNfL was regarded as a useful tool in the differential diagnosis, monitoring, and prognosis of neurological diseases. Previous studies have found that patients with amyotrophic lateral sclerosis, multiple sclerosis, Alzheimer's disease, frontotemporal dementia, Parkinson's disease, and Huntington's disease [2], as well as those with small vessel disease [17, 18], showed greater pNfL levels. At the same time, numerous studies have also shown that pNfL levels are related to cognitive dysfunction and dementia [2, ]. Our team has previously made clear the relationship between pNfL levels and cognitive impairment after anterior circulation stroke [16], but it is unclear whether it is related to posterior circulation. The posterior circulation accounts for around 20–25% of all acute strokes [20]. Strokes in the posterior circulation region have been proven in recent investigations to cause varying degrees of cognitive impairment. The cerebellum was involved in cognitive and emotional control [21]. Brain stem lesions mainly showed executive function and attention disorders [22, 23], thalamic lesions could result in a variety of cognitive problems [24]. Patients with isolated occipital stroke had cognitive impairment. Occipital stroke combined with lesions in the parahippocampal gyrus or corpus callosum pressure was associated with cognitive decline in patients with posterior cerebral artery stroke [25]. Therefore, it is necessary to pay attention to the cognitive impairment after a posterior circulation stroke. As far as we know, it is the first study to investigate the relationship between cognitive impairment and pNfL levels after posterior circulation stroke.

NfL is an intermediate filament protein that is heavily produced in axons and is a component of the cytoskeleton of neurons. NfL levels in the brain rise after axonal injury and neurodegeneration [26]. The identification and quantification of axonal damage could help to make an evaluation after the stroke. Animal experiments suggested that pNfL levels were significantly negatively correlated with cognitive function [26]. Previous studies have suggested that pNfL levels are related to cognitive change [11, 12, 26]. Osborn et al. [27] suggested that not only CSF NfL but also pNfL were related to cognition. According to a recent study, pNfL levels were related to cognitive function and could be used as a predictor of ongoing functional recovery and development [11]. Our study also showed that patients with PSCI had higher levels of pNfL, which are considerably inversely associated with cognitive function. This is in line with the findings mentioned above. The potential pathophysiology behind pNfL in stroke should be taken into consideration. The brain areas supplied by the posterior circulation are connected with the relevant areas of the cerebral cortex involved in advanced cognitive function through pathways, and stroke can lead to the degeneration of neurons and interruption of connection pathways, thus affecting cognitive function. The increase of pNfL levels reflects secondary neurodegeneration caused by a stroke, as well as alterations in the white matter and other neurodegenerative processes.

PNfL levels and stroke severity judged by the NIHSS and infarct volume measured by DWI are significantly related in our research; these findings are consistent with multiple earlier investigations [28–30]. Previous research has shown that NFL concentration fluctuated dynamically with time and that the acute phase sNfL level increased as the blood sampling delayed [30]. Our research also found that the pNfL level increased with the time from symptom onset to blood sampling increasing. However, there was no substantial difference in the time it took to sample blood between the two groups. It is similar to a previous study that pNfL was positively associated with age [31]. The PCSI group had higher homocysteine which was consistent with a previous study [32].

For the first time, we find that pNfL can predict cognitive damage following a posterior circulation stroke. Our research may contribute to putting pNfL into clinical practice. Based on our results, pNfL might be used in clinical practice as a screening biomarker to find patients at high risk for cognitive impairment after posterior circulation stroke. However, there are some limitations in our research. First, because the sample size for an observational research was relatively small, studies in larger patient cohorts are needed to confirm our observations. Second, the pNfL level was only measured once (within 48 h of onset). As a result, we were unable to determine how pNfL changed over time after a stroke or the relationship between the changes in pNfL over time and PSCI. Third, the plasma level of NfL rather than the CSF level was measured. It was not clear whether the variation in plasma levels was reflected in CSF although it had been reported that there was a significant correlation between CSF, NfL, and pNfL [27].

## 5. Conclusion

Our research revealed that higher pNfL levels within 48 h were correlated with 90-day cognitive impairment following acute ischemic stroke, even after clinically relevant influencing factors have been taken into account. Our research found biomarkers that could be used to diagnose cognitive deterioration following a posterior circulation stroke. This biomarker is not the only one, which needs further research to verify.

## Figures and Tables

**Figure 1:** Plasma neurofilament light chain (pNfL) concentration was substantially greater in the poststroke cognitive impairment (PSCI) group in comparison with the non-PSCI group.

**Figure 2:** (a–d) The relationship between the National Institutes of Health Stroke Scale (NIHSS), infarction volume (ml), the blood sampling time (h), the Montreal cognitive assessment (MOCA), and plasma NfL levels was analyzed using Spearman correlation.

**Figure 3:** Receiver operating characteristic curve for the plasma neurofilament light chain. AUC, area under the curve.

**Table 1:** Baseline characteristics of the participants.

Factors	Total	PSCI	Non-PSCI	*p*
Overall rate, *n* (%)	264 (100)	101(38.30)	163 (61.70)	
Sex, male, *n* (%)	157 (59.47)	55 (54.46)	102 (62.60)	0.191
Age (y), median(IQR)	65 (51–73)	68 (56.50–76.50)	62 (49–71)	0.005
Education level, <6 years, *n* (%)	76 (28.78)	27 (26.73)	49 (30.06)	0.562
Vascular risk factors, n (%)				
Hypertension	144 (54.54)	61 (60.39)	83 (50.92)	0.133
Diabetes mellitus	73 (27.65)	29 (28.71)	44 (26.99)	0.762
Hyperlipidemia	52 (19.70)	27 ( 26.73)	25 (15.34)	0.024
Atrial ﬁbrillation	32 (12.12)	12 (11.88)	20 (12.27)	0.925
Smoking	97 (36.74)	33 (32.67)	64 (39.26)	0.280
Drinking	62 (23.48)	19 (18.81)	43 (26.38)	0.159
NIHSS, median (IQR)	5 (3–8)	7 (3–10)	4 (2–7)	0.001
Infarct volume (ml), median (IQR)	12.87 (7.76–19.19)	18.06 (12.56–24.14)	11.05 (3.30–15.35)	<0.001
TOAST classification, *n* (%)				0.192
Large-artery atherosclerosis	151 (57.20)	64 (63.37)	87 (53.37)	
Cardioembolism	44 (16.67)	16 (15.84)	28 (17.18)	
Small vessel occlusion	23 (8.71)	9 (8.91)	14 (8.59)	
Other cause	18 (6.82)	7 (6.93)	11 (6.75)	
Undetermined	28 (10.61)	5 (4.95)	23 (14.11)	
Blood sampling time (h), median (IQR)	26.00 (15.00–37.00)	28.00 (19.50–40.00)	25.00 (14.00–36.00)	0.103
Plasma NfL (pg/mL), median (IQR)	38.68 (24.61–53.85)	49.54 (40.00–78.59)	30.12 (19.88–43.61)	<0.001
HbA1c (%), median (IQR)	5.90 (5.5–7.30)	5.90 (5.60–7.55)	5.90 (5.40–7.00)	0.259
Hs-CRP (mg/L), median (IQR)	3.33 (2.16–4.78)	3.20 (2.56–4.72)	3.48 (2.12–4.84)	0.871
Homocysteine (umol/L), median (IQR)	15.54 (11.32–21.76)	16.45 (12.32–22.91)	15.14 (10.13–21.70)	0.042
MOCA, median (IQR)	26.00 (23.25–27.00)	22.00 (19.00–24.00)	26.00 (26.00–28.00)	<0.001

PSCI, poststroke cognitive impairment; IQR, interquartile range; NIHSS, National Institutes of Health Stroke Scale; TOAST, Trial of ORG 10172 in Acute Stroke Treatment; Hs-CRP, high-sensitivity C-reactive protein; MOCA, Montreal Cognitive Assessment.

**Table 2:** Logistic regression analysis for the association of pNfL with PSCI.

Variables	OR	95% CI	*p*
Unadjusted pNfL	1.044	1.031–1.059	<0.001
Model 1 pNfL	1.044	1.030–1.058	<0.001
Model 2 pNfL	1.035	1.019–1.051	<0.001

pNfL, plasma neurofilament light chain. Model 1 is adjusted for age, gender, and educational level. Model 2 is adjusted for Model 1 and baseline NIHSS score, infarct volume, and TOAST classification.

## Data Availability

The datasets supporting the conclusions are available from the corresponding author on reasonable request.
